The article "Diagnosis of Arrhythmia for Patients with Occult Coronary Heart Disease Guided by Intracavitary Electrocardiogram under Data Mining Algorithm" was published in 2021. Journal: J Healthc Eng.

# Diagnosis of Arrhythmia for Patients with Occult Coronary Heart Disease Guided by Intracavitary Electrocardiogram under Data Mining Algorithm

**DOI:** 10.1155/2021/1640870

**Published:** 2021-09-11

**Authors:** Gang Wang, Li Luo, Xia Zhao

**Affiliations:** ^1^Department of Geriatrics, Lianshui County People's Hospital, Lianshui 223400, China; ^2^Department of Cardiology, The Affiliated Huai'an Hospital of Xuzhou Medical University and The Second People's Hospital of Huai'an, Huai'an 223002, China; ^3^Department of Cardiology, The Second Affiliated Hospital of Jiaxing University, Jiaxing, Zhejiang 314000, China

## Abstract

The objective of this study was to explore the application value of intracavitary electrocardiogram- (IEGM-) guided diagnosis of occult heart disease and conventional electrocardiogram (EGM) in the diagnosis of occult coronary heart disease (CHD) based on the classification and regression tree (CART) mining algorithm, hoping to provide a more effective basis for clinical diagnosis of the occult CHD. In this study, 100 patients with occult CHD admitted to our hospital from February 2016 to December 2020 were selected as the research objects. Based on the random number table method, 100 patients were randomly rolled into two groups, each with 50 cases. The patients diagnosed with conventional ECG were set as the control group, and patients in the experimental group were diagnosed with IEGM under the data mining algorithms. The diagnostic effects of the two groups were compared. The results showed that the processing effect of the CART algorithm (94%) was much better than that of the multiple linear regression algorithm (78%) and the random forest algorithm (69%) (*P* < 0.05), the agreement between the results of the experimental group and the results of coronary angiography (80%) and Kappa (0.7) was higher than those of the control group (55%, 0.45), and the difference was statistically significant (*P* < 0.05). In addition, the sensitivity (93%) and accuracy (80%) of the experimental group were obviously higher than those of the control group (62% and 55%), and the differences were remarkably significant (*P* < 0.05). In conclusion, the consistency ratio of the IEGM examination was higher, showing high accuracy; the intracavitary examination was invasive, so IEGM was not recommended when the diagnosis result of the examination may cause more harm than good.

## 1. Introduction

The economic, cultural, and technological development of today's society is quite rapid, including the medical technology. With the development of society, it is not only people's living standards that have been improved, but the incidence of various diseases has also increased, which has had a great impact on people's lives and health, including the hidden coronary heart disease (occult CHD) [1, 2]. The pathogenesis of coronary heart disease (CHD) is mainly due to coronary artery stenosis that causes the circulatory system to not provide enough blood to the body, which indirectly leads to myocardial dysfunction. CHD can be said to be a common disease with a high clinical incidence, and its occurrence trend is also increasing year by year with time [3, 4]. The occult CHD, also known as painless myocardial ischemia, is a special type of CHD [5]. Most people with occult CHD are middle-aged or older. Simply speaking, it means that there is no obvious clinical manifestation. However, myocardial ischemia and coronary atherosclerosis can be found under the relevant examinations of electrocardiogram (EGM), dynamic EGM, and cardiac color Doppler ultrasound [6, 7].

The article "Diagnosis of Arrhythmia for Patients with Occult Coronary Heart Disease Guided by Intracavitary Electrocardiogram under Data Mining Algorithm" was published in 2021. Journal: J Healthc Eng.

Since the diagnosis of occult CHD is relatively difficult, the clinically frequently used diagnostic method is EGM, including dynamic EGM and stress test EGM. However, the operations of these two examination methods are more complicated and difficult to use, which makes it difficult for their clinical applications to be popularized. Although selective coronary angiography can improve the clinical detection rate, it is an invasive operation. To a certain extent, the patient's tolerance must be taken into account, so it will lead to high clinical misdiagnosis and missed diagnosis [8, 9]. As a mapping technique that places electrode catheters in different parts of the heart to record cardiac indicators, intracavitary electrocardiogram (IEGM) uses the guide wire in the catheter as the electrode and monitors the changes in the EGM P wave that occur during catheter placement to determine the tip of the catheter location [10]. The IEGM is a new cutting-edge positioning method for peripherally inserted central venous catheters (PICC), which can effectively dilute high-concentration and irritating drugs, protecting the blood vessels and relieving patients' pain [11]. But there are still limitations in the application of this technology. It is difficult to distinguish between atrial and ventricular waves by observing the results of IEGM alone, and the extracavitary electrocardiogram has to be required during the analysis process.

With the widespread application of intelligent algorithms in the medical field, people also try to combine intelligent algorithms with intracavitary electrocardiogram inspection methods to obtain a good diagnosis of occult coronary heart disease. However, there are relatively few researches on this type. Data mining algorithm is a set of heuristics and calculations to create a data mining model based on data. The provided data were analyzed firstly using the algorithm, and a specific type of pattern and trend would be found to create the model [12]. This study was intended to explore the application value of IEGM based on data mining algorithms and conventional EGM in diagnosis of occult CHD, hoping to provide a more effective basis for its clinical diagnosis.

The article "Diagnosis of Arrhythmia for Patients with Occult Coronary Heart Disease Guided by Intracavitary Electrocardiogram under Data Mining Algorithm" was published in 2021. Journal: J Healthc Eng.

## 2. Methods

### 2.1. Research Objects

100 patients with occult CHD admitted to the hospital from February 2016 to December 2020 were selected as the research objects. There were 52 males and 48 females, aged 45–72 years (with an average age of 56.1 ± 3.8 years). Based on the random number table method, 100 patients were randomly rolled into two groups, each with 50 cases. The patients diagnosed with conventional ECG were set as the control group, and patients in the experimental group were diagnosed with IEGM under the classification and regression tree (CART) data mining algorithm. The diagnostic effects of the two groups were compared. The general clinical data of the two groups of patients (Table 1) revealed that the comparison was not statistically significant (*P* > 0.05) but comparable, suggesting the feasibility of this experiment. This study had been reviewed by the Ethics Committee of our hospital.

The inclusion criteria were given as follows: patients over 18 years, patients who suffered with coronary atherosclerosis and myocardial ischemia without pain, patients with at least one coronary artery stenosis ≥ 50% diagnosed by selective coronary angiography, and patients who were informed about the study and signed the informed consent forms.

The exclusion criteria were defined as follows: patients with malignant tumor disease; patients with severe immunization and infectious diseases; patients with cognitive impairment and unable to complete the study; patients with pacemakers and 24 h dynamic EGM; patients who had been diagnosed with atrial fibrillation, supraventricular tachycardia, pulmonary heart disease, and other heart diseases that affected the shape of the *P* wave; patients who were prone to muscle tremor, such as hyperthyroidism; and patients whose basic EGMs were difficult to clearly identify.

### 2.2. Research Methods

The conventional EGM was performed as for patients in the control group. The posture of the patient was guided by professional person so that they were relaxed enough. The specific operation process is shown in Figure 1.

The IEGM was performed for patients in the experimental group, and the involved materials and instruments included catheter material (1.9 F PICC catheter with guide wire), EGM monitor (PHILPS MP20), IEGM wire, EGM electrode clips, and conversion adapter.

The article "Diagnosis of Arrhythmia for Patients with Occult Coronary Heart Disease Guided by Intracavitary Electrocardiogram under Data Mining Algorithm" was published in 2021. Journal: J Healthc Eng.

The specific operation process is shown in Figure 2: the catheter placement was performed by the static therapy specialist nurses in accordance with the PICC catheter placement in the hospital and the standardized operating procedures for IEGM positioning.

### 2.3. Analysis Model of Data Mining Algorithm

In this study, the classification and regression tree (CART) mining algorithm in the data mining algorithm was adopted to build the analysis model. The CART is commonly used to process continuous data, and heuristic methods are used to minimize the quadratic variance of each node, thus completing the division of the input space [13].

The *n*^*th*^ variable *x*^*n*^ and its value *m* were selected as the segmentation variable and segmentation point, respectively, and two regions *Q*_1_ and *Q*_2_ were defined as shown in the following equations:

(1) $$\begin{array}{c} Q_{1}\left(n,m\right)=\left\{x|x^{n}\leq m\right\}, \end{array}$$

(2) $$\begin{array}{c} Q_{2}\left(n,m\right)=\left\{x|x^{n}>m\right\}. \end{array}$$

Then, the best segmentation variable *n* and segmentation point *m* were found out, and the specific solution process is shown as follows:

(3) $$\begin{array}{c} \underset{n,m}{\min}\left[\underset{z_{1}}{\min}\underset{x_{1}\in Q_{1}\left(n,m\right)}{\sum }{\left(y_{i}-z_{1}\right)}^{2}+\underset{z_{2}}{\min}\underset{x_{1}\in Q_{2}\left(n,m\right)}{\sum }{\left(y_{i}-z_{2}\right)}^{2}\right], \end{array}$$

(4) $$\begin{array}{c} Z_{1}=\mathrm{ave}\left(y_{i}|x_{i}\in Q_{1}\left(n,m\right)\right), \end{array}$$

(5) $$\begin{array}{c} Z_{2}=\mathrm{ave}\left(y_{i}|x_{i}\in Q_{2}\left(n,m\right)\right). \end{array}$$

In the above equation, *x*_*i*_, *y*_*i*_, and *Z*_*1*_ referred to independent variable, dependent variable, and optimal solution, respectively. In this study, the CART mining algorithm was adopted to process a large amount of particle information in the IC-EGM detection to increase the accuracy of the inspection results.

### 2.4. Observation Indicators

Two experienced and highly qualified physicians were invited to judge all examination results. The result of coronary angiography was undertaken as the gold standard to compare the consistency of the results. The sensitivity, specificity, accuracy, positive predictive value, and negative predictive value were calculated based on the test results. The calculation standard of curative effect was shown in Table 2.

### 2.5. Statistical Methods

The SPSS22.0 was adopted for data entry, sorting, and statistical analysis. The enumeration data were compared using *χ*^2^ test; and the measurement data were compared using *t*-test. The multiple sample means were compared with the analysis of variance. The LSD method was used when the variance was uniform, and the Dunnett T3 method was used when the variance was uneven. *P* < 0.05 indicated that the difference was statistically significant. Kappa test was performed on the consistency ratio between the examination result and the coronary angiography results in two groups. When Kappa > 0.75, the consistency rate between the two results was high; when 0.4 ≤ Kappa < 0.75, the consistency rate was normal; and when Kappa < 0.4, the consistency rate was low.

The article "Diagnosis of Arrhythmia for Patients with Occult Coronary Heart Disease Guided by Intracavitary Electrocardiogram under Data Mining Algorithm" was published in 2021. Journal: J Healthc Eng.

## 3. Results

### 3.1. Comparison on IC-EGM Processing Effect

In the research process, the effect of multiple linear regression algorithm, random forest algorithm, and CART algorithm were compared on IC-EGM processing. The final diagnosis result was undertaken as the gold standard to compare the accuracy of the diagnosis result. The results showed that the accuracy of the IC-EGM detection results processed by the multiple linear regression algorithm was 78%, and that was 69% for the random forest algorithm and 94% for CART algorithm. The comparison revealed that the processing effect of the CART algorithm was much better than the multiple linear regression algorithm and the random forest algorithm (*P* < 0.05), as shown in Figure 3.

### 3.2. Comparison of EGM Results of Healthy Person and Patients with CHD

Figure 4(a) shows the standard EGM results of normal people, and Figure 4(b) shows the EGM manifestations of patients with CHD. Comparison of the two EGM results revealed that the trend of *P* wave in the EGM of patients with CHD weakened and decreased, with basically disappeared *Q* wave and lower position of ST segment compared with the results of normal people, showing an oblique ST segment decline, inverted T wave, and basically normal QRS band.

### 3.3. Comparison on the Diagnosis Results of the ECG of the Two Groups of Patients

Figure 5 shows the test results under a conventional EGM. It disclosed that there were 31 patients with positive test results and 19 with negative results in the control group. The comparison between the positive rate and the negative rate in this group of patients suggested that the positive rate was higher than the negative rate, and the difference was statistically significant (*P* < 0.05).  Figure 6 shows the test results under IEGM. It revealed that there were 46 patients with positive test results and 4 patients with negative results in the experimental group. The comparison showed that the positive rate was higher than the negative rate, and the difference was statistically obvious (*P* < 0.05).

The article "Diagnosis of Arrhythmia for Patients with Occult Coronary Heart Disease Guided by Intracavitary Electrocardiogram under Data Mining Algorithm" was published in 2021. Journal: J Healthc Eng.

### 3.4. Comparison on the Consistency between Examination Results and the Coronary Angiography Results between Two Groups

Table 3 shows the statistics of the results in the control group. It disclosed that in the control group, there were 28 cases with the consistent results between the conventional EGM and the coronary angiography, including 21 positive cases and 7 negative cases. Therefore, the consistency ratio was 55%.  Table 4 shows the statistics of the results in the experimental group. It was clear that in the experimental group, there were 42 cases with the consistent results between the IEGM examination and the coronary angiography, including 39 positive cases and 3 negative cases, so the consistency ratio was 80%. The consistency ratios between the examination results and the coronary angiography results and the Kappa test results were compared, and the results are illustrated in Figure 7. The results in the experimental group were higher than those of the control group, showing statistically great difference (*P* < 0.05), indicating the IEGM examination showed higher consistency, so the accuracy was higher.

### 3.5. Comparison on Diagnostic Effect of Two Different Examinations

The diagnostic effect between the experimental group and the control group after examination was compared, as illustrated in Figure 8. The diagnostic sensitivity and accuracy in the experimental group were 93% and 80%, respectively, while those in the control group were 62% and 55%, respectively. Thus, the diagnostic sensitivity and accuracy in the experimental group were much higher in contrast to those in the control group, and the difference was statistically great (*P* < 0.05). The specificity in control group was slightly higher in contrast to the experimental group, showing not statistically obvious difference (*P* > 0.05).

## 4. Discussion

As the quality of life of people in today's society has been greatly improved, the food, clothing, housing, and transportation have been greatly improved, especially in terms of diet [14]. As the pace of people's lives continues to accelerate, the dietary structure, types of diet, and dietary styles have become diversified. In addition, the diseases have become diversified, and the incidence of various diseases has increased year by year [15]. At present, the incidence of CHD is showing a slow upward trend. CHD is mainly due to the vascular blockage or stenosis caused by coronary atherosclerosis in patients. The blood circulation in the patient's blood vessels is blocked, so that the normal function is affected, and then convulsions occur, which eventually leads to myocardial hypoxia and ischemia [16]. If the patient cannot be treated in time after the onset of the CHD, it will lead to sudden death and endanger the patient's life. According to clinical studies, the types of CHD are relatively diverse, mainly manifested as angina pectoris, myocardial infarction, and occult [17, 18]. The occult CHD has a particularly high clinical incidence, and it is mainly in the elderly. As a CHD lacking relevant clinical symptoms, occult CHD is also a cardiovascular event with higher risk factors, and it is affected by no obvious clinical symptoms, so the missed diagnosis rate is high, which brings great hidden dangers to the life safety of patients [7, 19].

The article "Diagnosis of Arrhythmia for Patients with Occult Coronary Heart Disease Guided by Intracavitary Electrocardiogram under Data Mining Algorithm" was published in 2021. Journal: J Healthc Eng.

In order to effectively improve the diagnostic accuracy of patients with occult CHD, the current clinical diagnosis is mainly based on EGM, which greatly improves the clinical diagnosis effect of patients. However, there are still some shortcomings in conventional EGM diagnosis. Therefore, the conventional EGM was adopted to diagnose 50 patients with suspected occult CHD in the control group, and the IEGM based on data mining algorithms was adopted to diagnose and analyze the other 50 patients in the experimental group in this study. In addition, the consistency between the examination results of the coronary angiography results was calculated and compared between two groups. According to the diagnosis results, the diagnostic sensitivity and accuracy in the experimental group were higher than those in the control group, and the specificity was basically similar, indicating that the IEGM showed higher diagnostic accuracy in occult CHD patients clinically. The application of IEGM not only is applicable in the diagnosis of heart disease, but also can assist the positioning of the PICC catheter to reduce the occurrence of neonatal complications. Many experts have discussed the impacts of IEGM-assisted positioning technology on the complications of PICC in neonates. Research results have shown that in the process of neonatal PICC catheterization, the use of IEGM-assisted positioning can reduce catheter-related complications [20, 21]. There are also research experts selected by typical EGMs of different parts of the heart cavity and their evolutionary characteristics as the guidance to replace the X-ray fluoroscopy for bedside temporary endocardial pacing of 22 cases; the success rate was 100%, the average operation time was 18 minutes, the average pacing from intubation to the right ventricle was 48 seconds, and the average pacing threshold was 0.72 V; there were no other complications except for electrode dislocation. Compared with 30 cases of temporary pacing under traditional fluoroscopy, there was no significant difference in various indicators. The results showed that cardiac IEGM-guided bedside pacing was a first-aid measure that was reliable, easy to operate, safe, practical, and easy to popularize [22]. The retrospective analysis in this study suggested that the high-frequency wavelet part had to be filtered in the conventional EGM examination to keep the waveform smooth and clear. As a result, the high-frequency signal cannot be fully displayed in the conventional EGM examination result, which in turn caused some high-frequency signals to be lost in the EGM result. Therefore, conventional EGM examination is only suitable for patients with a wide range of myocardial ischemic necrosis, and occult CHD patients with mild myocardial ischemia cannot show typical EGM signs of CHD [23].

The article "Diagnosis of Arrhythmia for Patients with Occult Coronary Heart Disease Guided by Intracavitary Electrocardiogram under Data Mining Algorithm" was published in 2021. Journal: J Healthc Eng.

Lupi et al. (2016) [24] found that IEGM is more sensitive than the extracavitary electrocardiogram in reflecting the myocardial ischemia during percutaneous transluminal coronary angioplasty (PT-CA). Drago et al. (2018) [25] suggested that the change of IEGM into the ST segment can reflect the viability of the residual myocardium to a certain extent. Moreover, some people have studied and proposed that IEGM can detect the viable myocardium at the infarcted area of patients with acute myocardial infarction and predict the postoperative efficacy of coronary intervention. Therefore, the clinical application value of IEGM is very high [26].

## 5. Conclusion

Based on the above research results, it could be concluded that the sensitivity and accuracy of IEGM results based on data mining algorithm analysis were higher than those of conventional EGM, and it showed very high application value in diagnosis of related diseases and in the guidance for treatment of related diseases, reflecting the good development prospects of IEGM in the clinical field. However, the intracavitary examination was invasive, so it was not recommended when the diagnosis result of the examination may cause more harm than good.

## Figures and Tables

**Figure 1:** The specific operation process of conventional EGM.

**Figure 2:** The specific operation process of IEGM.

**Figure 3:** Comparison on diagnosis accuracy of different algorithms. *Note*. ^*∗*^*P* < 0.05.

**Figure 4:** Comparison of EGM results of healthy person and patients with CHD. (a) The standard EGM results of normal people and (b) the EGM manifestations of patients with CHD.

**Figure 5:** EGM results of patients in the control group. *Note*. ^*∗*^*P* < 0.05.

**Figure 6:** IEGM results of patients in the experimental group. *Note*. ^*∗*^*P* < 0.05.

**Figure 7:** Comparisons on consistency ratio and Kappa results. *Note*. ^*∗*^*P* < 0.05.

**Figure 8:** Comparison on diagnostic effect of two different examinations. *Note*. ^*∗*^*P* < 0.05.

The article "Diagnosis of Arrhythmia for Patients with Occult Coronary Heart Disease Guided by Intracavitary Electrocardiogram under Data Mining Algorithm" was published in 2021. Journal: J Healthc Eng.

**Table 1:** The general clinical data of the two groups of patients.

Group	Gender		Age range (years)	Average age (years)
	Males (*n* = 52)	Females (*n* = 48)		
Experimental group (50 cases)	27	23	45–70	56.4 ± 3.1
Control group (50 cases)	25	25	45–71	55.8 ± 3.8
*χ* ^2^	3.182	2.198	2.391	2.981
*P*	0.121	0.081	0.096	0.101

**Table 2:** The calculation standard of curative effect.

Indicators	Calculation methods
Sensitivity	Number of true-positive cases/(number of true-positive cases + number of false-negative cases) × 100%
Specificity	Number of true-negative cases/(number of true-negative cases + number of false-positive cases) × 100%
Accuracy	EGM result/coronary angiography result × 100%

**Table 3:** The statistics of the results in the control group.

Control group	Coronary angiography		Total
	Positive	Negative	
Positive	21	10	31
Negative	12	7	19
Number of consistent results	21	7	28

**Table 4:** The statistics of the results in the experimental group.

Experimental group	Coronary angiography		Total
	Positive	Negative	
Positive	39	7	46
Negative	1	3	4
Number of consistent results	39	3	42

## Data Availability

The data used to support the findings of this study are available from the corresponding author upon request.
